The article "AIB1 Cooperates with ERα to Promote Epithelial Mesenchymal Transition in Breast Cancer through SNAI1 Activation" was retracted in 2021. Reasons: manipulated images; duplicated images; original data or images not available; unreliable data.

# AIB1 Cooperates with ERα to Promote Epithelial Mesenchymal Transition in Breast Cancer through SNAI1 Activation

**DOI:** 10.1371/journal.pone.0065556

**Published:** 2013-06-07

**Authors:** Miao Wang, Feng Zhao, Shujing Li, Alan K. Chang, Zhaojun Jia, Yixuan Chen, Feihong Xu, Hongming Pan, Huijian Wu

**Affiliations:** School of Life Science and Biotechnology, Dalian University of Technology, Dalian, China; Philipps University, Germany

## Abstract

Epithelial Mesenchymal Transition (EMT) plays a major role in cancer metastasis. Several genes have been shown to play a role in EMT, and one of these is Amplified-in-breast cancer 1 (*AIB1*), which has oncogenic function and is known to be amplified in breast cancer. However, the role of AIB1 in EMT remains largely undefined at the molecular level. In this study, the effect of AIB1 overexpression on the EMT of the breast cancer cell line T47D was investigated. Overexpression of AIB1 disrupted the epithelial morphology of the cells. At the same time, the cells displayed a strong metastasis and reduced level of the epithelial marker E-cadherin. In contrast, knockdown of AIB1 in T47D cells increased cell-cell adhesion and produced weak metastasis, as well as a higher level of E-cadherin expression. We proposed that the regulation of EMT by AIB1 occurred through the action of the transcription factor SNAI1, and demonstrated that such interaction required the participation of ERα and the presence of ERα-binding site on SNAI1 promoter. The expression level of E-cadherin and the extent of cell migration and invasion in SNAI1-knocked down T47D cells that overexpressed AIB1 were similar to those of T47D cells that did not overexpress AIB1 and had no SNAI1 knockdown. Taken together, these results suggested that AIB1 exerted its effect on EMT through its interaction with ERα, which could directly bind to the ERα-binding site on the SNAI1 promoter, allowing the AIB1-ERα complex to promote the transcription of SNAI1 and eventually led to repression of E-cadherin expression, consistent with the loss of E-cadherin being a hallmark of EMT.

## Introduction

Breast cancer is the most common malignancy among women, and it is the second leading cause of death among women having cancer [1]. Breast cancer mortality is largely attributed to metastasis. Despite its clinical relevance, research on the molecular mechanisms of epithelial mesenchymal transition (EMT) has not been extensively pursued, partly due to a lack of appropriate experimental models and difficulties in identifying metastasis-specific regulators and mediators [2].

EMT is considered as an important step in metastasis, during which non-motile, polarized epithelial cells dissolve their cell-cell junctions and convert into individual and motile mesenchymal cells [3], [4]. Cells undergoing EMT have several prominent features, including a change in cell morphology from round compact epithelial shape to spindle-scattered mesenchymal phenotype accompanied by the loss of E-cadherin [5], [6]. However, some cells undergoing partial EMT instead of complete EMT, and these cells retain some of the characteristics of epithelium and also display features of mesenchymal cells, a phenomenon which is recognized as partial EMT [7]. Several transcription factors are known to play a central role in the activation of EMT by acting as EMT inducers. These transcription factors include SNAI1 (Snail), SNAI2 (Slug) and ZEB1, all of which interact with the proximal E-boxes of E-cadherin promoter [8]. Therefore, understanding the regulation of these transcriptional factors would provide important insights into the molecular mechanisms implicated in breast tumor metastasis.

Amplified-in-breast cancer 1 (AIB1 also known as SRC-3, ACTR, p/CIP, RAC3, TRAM1 and NCOA3) is a member of the p160 family, which also contains SRC-1 and SRC-2 [9], [10], [11], [12], [13], [14], [15], [16]. AIB1 is a transcriptional coactivator that promotes the transcriptional activity of multiple nuclear receptors such as estrogen receptors α (ERα) and other transcription factors such as Sp1, AP-1 and E2F1 [17], [18], [19]. ERα is a well-known estrogen (E2)-dependent receptor that plays a critical role in breast cancer development, and its functions are primarily mediated by AIB1 [9], [10], [13], [14].

Although the role of AIB1 in the proliferation of primary tumor in the mammary gland is well established, a role for this oncogenic coregulator in tumor cell motility and metastasis has been elucidated only recently. In the nucleus, AIB1 is essential for proteolytic breakdown of the extracellular matrix by matrix-metalloproteinases, a process which enables primary tumor cells to invade the surrounding stroma [20], [21]. At the plasma membrane, an exon-4-truncated isoform of AIB1 (AIB1Δ4) lacking the N-terminal bHLH domain (which contains a nuclear localization signal) serves as a signaling adaptor for the epidermal growth factor, focal adhesion kinase and c-Src signal transduction pathway, all of which are implicated in metastasis and invasion [22]. Together, these studies underscore a pivotal role of AIB1 not only as a proto-oncogene, but also as a prometastatic factor during the early stages of metastasis [23]. However, the contribution of AIB1 in the regulation of tumor metastasis and the underlying mechanism of this process is largely unknown.

We have previously shown that the AIB1 is required for breast cancer cell proliferation and demonstrated that its transcriptional activity is up-regulated by phosphorylation and down-regulated by sumoylation, and identified PIAS1 as the SUMO E3 ligase that can enhance the sumoylation of AIB1, thereby down-regulating AIB1 transcriptional activity [24], [25]. In this study, we used a combined molecular and cellular approach to characterize the role of AIB1 in EMT. We showed that cooperation between AIB1 and ERα raised SNAI1 expression and repressed E-cadherin transcriptional activation, resulting in the promotion of EMT in breast cancer cells.

## Results

### AIB1 is Associated with Cell-cell Adhesion in Breast Cancer Cells

Elevated level of AIB1 is frequently associated with distant metastasis, high tumor grade and poor prognosis, especially for breast tumor. The morphologies of three estrogen receptor alpha-positive (ERα+) human breast cancer cell lines (ZR-75-1, MCF-7 and T47D) with different invasive capabilities were analyzed and compared. The order of increasing invasiveness for the three cell lines was ZR-75-1<MCF-7<T47D. Thus T47D cells showed the least cell-cell contact compared to the other two cell lines, whereas ZR-75-1 cells exhibited the most compact colonies (Fig. 1A). Analysis of the protein levels of AIB1 and ERα in these cell lines showed an increased level of AIB1 in T47D cells, but no obvious change in the level of ERα was detected among the three cell lines (Fig. 1B). This implied that AIB1, which is often highly expressed in breast cancer cells, might play a role in controlling the morphological characteristics of these cells well as the extent of their cell-cell contact.

**Figure 1:** AIB1 regulates the morphologies of breast cancer cells. (A) Light microscopic images showing the morphology of different breast cancer cells. (B) Expression levels of AIB1, ERα and E-cadherin in different breast cancer cells as detected by western blot analysis. Cell extracts were prepared from the different cell lines and probed with specific antibody against AIB1, ERα and E-cadherin or β-actin. (C) Light microscopic images showing EMT morphological changes induced in T47D cells after treatment with EGF (50 ng/ml) or E2 (20 nM) for 24 h. (D) Western blot analysis showing the levels of AIB1, ERα, E-cadherin and β-actin expressions in T47D cells after treatment with EGF or E2. (E) Coimmunoprecipitation showing AIB1 and ERα complex increased after treatment with EGF or E2. T47D cells treated without or with EGF (50 ng/ml) or E2 (20 nM) for 24 h were subjected to immunoprecipitation with anti-AIB1 or control IgG antibodies, followed by western blot analysis with anti-ERα and anti-AIB1 antibodies. (F) Light microscopic images showing T47D cells without or with AIB1 knockdown (shAIB1#1 and shAIB1#2), ERα knockdown (shERα) or both AIB1 and ERα knockdown. Cells were treated with the corresponding iRNA and then plated out in 50-mm dishes and incubated for 3 days before observing. (G) The cells from (F) were counted and plotted as percentage of clustered or scattered cells relative to total number of cells (400–500). (H) Western blot analysis showing the levels of AIB1, ERα, E-cadherin and β-actin proteins in T47D cells from (F).

Previous study has shown that EGF signal pathways can reduce cell-cell contact and induce metastasis [26]. Treatment of T47D cells with EGF leads to activation of MAPK pathway, and the resulting phosphorylation of MAPK enhances the transcriptional activity of AIB1 [27]. We also observed changes in the morphology of T47D cells after treatment with EGF. The cells became scattered, with loss of close cell-cell junctions and formation of spindle-shaped appearance, which are morphological changes that are reminiscent of the cells belonging to the mesenchymal lineage (Fig. 1C). In addition, these cells also showed reduced expression level of the critical epithelial protein E-cadherin (Fig. 1D). Treatment of T47D cells with E2 also induced mesenchymal morphology and reduced cell-cell contact. Most importantly, no significant upregulation of AIB1 and ERα expressions was observed when these cells were treated with EGF or E2 (Fig. 1D). Our previously study has shown that treatment of MCF-7 cells with E2 resulted in increased levels of phosphorylated AIB1 and enhancement of AIB1 transcriptional activity [24]. The interaction between AIB1 and ERα in T47D cells was demonstrated by coimmunoprecipitation experiments, and the result showed that formation of AIB1 and ERα complex increased almost two folds in EGF- or E2-treated cells compared to non-treated cells (Fig. 1E). This implied that AIB1 and ERα both might play a role in the loss of cell-cell contact and in the process that would ultimately cause the cells to become more scattered.

The effect of AIB1 or ERα on cell-cell contact was investigated by knocking down AIB1 or ERα or both AIB1 and ERα in T47D cells, and comparing the extent of cell-cell contact in these cells. Two shAIB1 sequences, shAIB1#1 and shAIB#2, were used to knock down AIB1 in the cells. Knocking down AIB1 with shAIB1#1 increased the overall proportion of clustered cells by 15%, whereas knocking down AIB1 with shAIB#2 increased it by 10%, relative to control cells. Knocking down ERα resulted in just 5% increase in the overall proportion of clustered cells (Figs. 1F&1G). Knocking down both AIB1 and ERα yielded the highest level of cell-cell contact, and increased the overall proportion of clustered cells by about 35% relative to control cells (Figs. 1F&1G). Knockdown of AIB1 increased the level of E-cadherin, a protein that is important for cell adhesion. Knockdown of AIB1 by shAIB1#1 increased the level of E-cadherin to more than two fold the level of control cells, whereas knockdown of AIB1 by shAIB1#2 increased the level of E-cadherin to about 1.5 fold the level of control cells. Since shAIB1#1 was more effective than shAIB1#2 at knocking down AIB1, all subsequent AIB1-knockdown experiments were conducted with shAIB1#1. Knockdown of ERα also caused some increase in the level of E-cadherin, but knockdown of both AIB1 and ERα caused the highest increase, almost three fold the level of control (Fig. 1H). These data implied that the role of AIB1 in cell-cell adhesion could in part be due to increases in the level of AIB1-ERα complex. Since AIB1 knockdown caused more disruption to cell-cell contact and higher increase in E-cadherin expression compared to ERα knockdown, part of the effect exerted by AIB1 on cell-cell contact in breast cancer cells might not be associated with ERα, the nature of which requires further investigation.

### AIB1 is Important in Breast Cancer Cells Motility and Invasion

Given that AIB1 could reduce cell-cell adhesion (Fig. 1 data), it then became important to know the relationship between AIB1 and cell motility and invasion in these tumor cells. AIB1 was therefore overexpressed in T47D cells and the effect its overexpression had on cell motility and invasion was determined by wound healing and transwell assays. Cells that overexpressed AIB1 showed faster wound healing with 50% more cells migrating through the uncoated membrane in the chamber compared to control cells that did not overexpress AIB1 (Fig. 2A). In addition, the migration of these cells through the Matrigel coated membrane (invasion assay) increased to 2.5 fold the number of control cells (Fig. 2B). Knockdown of AIB1 in T47D cells weakened the motility and invasiveness of the cells, as shown by wound healing and transwell migration and invasion assays (Fig. 2B). In order to confirm that the higher numbers of migrating and invading cells observed for cells that over expressed AIB1 were not a result of increase in cell proliferation caused by AIB1, we carried out MTT assay to compare differences in cell proliferation among control cells, T47D cells that over expressed AIB1 and those that had AIB1 knockdown. No significant differences in cell proliferation were observed among these different groups and no significant increases were detected at 24 h (Fig. 2C). This showed that the effect of AIB1 on cell proliferation within a 24-h period was insignificant, and therefore faster recovery of the wound achieved by cells that over expressed AIB1 and the stronger migration displayed by these cells compared to AIB1 knockdown cells were not due to cell proliferation caused by AIB1. This suggested that AIB1 might play an important role in tumor cell motility and invasion, and that this role is not contributed by its effect on cell proliferation.

**Figure 2:** AIB1 promotes cell motility and invasion in T47D cells. (A) Scratch wound-healing assay showing the effect of AIB1 on cell motility in T47D cells. Top panel: Images of T47D cells that were transfected with empty vector (pcDNA) or AIB1, and cells without (NC) or with AIB1 knockdown (shAIB1#1) before and after wound-healing assay. The cell layers were carefully wounded using a sterile 200-µl tip and then cultured for 24 h before evaluation. Bottom panel: Western blot analysis showing the levels of AIB1, ERα and β-actin expressions in pcDNA- or AIB1-transfected T47D cells, and of T47D cells without or with AIB1 knockdown. (B) Transwell migration and invasion assays showing the effect of AIB1 on cell motility and invasion ability in T47D cells. Images showing the migration and invasion of T47D cells that were transfected with empty vector (pcDNA) or AIB1, and of T47D cells without (NC) or with AIB1 knockdown (shAIB1#1). For NC group, the cells were transfected with a negative control scrambled shRNA synthesis DNA cloned into siRNA expression vector pRNAT carries GFP marker. Cell migration and invasion assays were performed in 24-well chambers without and with Matrigel, respectively. Cells (1000 per well) were transfected with GFP-AIB1 or just GFP (pEGFPC) and then transferred to the upper chamber. After 48 h of incubation, the numbers of migrating and invasive cells on the lower surface of the filter were counted under a fluorescent microscope. The bar graphs on the right of the images show the number of migrating and invading cells for each category of cells. (C) MTT assays showing the effect of AIB1 on cell proliferation in T47D cells. Cells were transfected as in (A) and then subjected to MTT assay within 24 hours.

### AIB1 Promotes EMT via Reduced Expression of E-cadherin

Increased motility and invasiveness shown by tumor cells are reminiscent of the events that occur during epithelial mesenchymal transition (EMT), and loss of E-cadherin expression is an essential event in EMT [26]. AIB1 might regulate cell motility and invasion through targeting the expression of E-cadherin, either at the protein or mRNA level or both. T47D cells that overexpressed AIB1 showed 50% reduction in the level of E-cadherin protein and 30% increase in the level of N-cadherin protein (a mesenchymal protein which is also important for EMT) compared to control cells (as determined by western blot), and similar results were also observed for MCF-7 cells that overexpressed AIB1 (Fig. 3A **).** Knocking down AIB1 in these cells resulted in the opposite effect. In the case of T47D cells, AIB1-knockdown resulted in about 50% increase in the level of E-cadherin and about 60% decrease in the level of N-cadherin compared to control cells (Fig. 3A). In the case of MCF-7 cells, knockdown of AIB1 produced very similar result as in T47D cells. A decreased level of E-cadherin and increased level of N-cadherin in both T47D and MCF-7 cells caused by AIB1 overexpression led to induction of mesenchymal cells morphology, as shown by immunofluorescence staining (Fig. 3C). Change in the level of E-cadherin mRNA paralleled with the change in level of E-cadherin protein, with about 40% less in cells that overexpressed AIB1 compared to control cells, as shown by real time PCR (Fig. 3D). However, reporter gene activity assay showed a much higher decrease in E-cadherin reporter activity in cells that over expressed AIB1 relative to control cells (Fig. 3E). At the same time, the level of E-cadherin mRNA in these cells also increased by about 30% (Fig. 3D), while the level of E-cadherin reporter activity increased almost by 100% over control cells (Fig. 3E). These data confirmed that the main effect AIB1 had on E-cadherin was on its gene transcription.

**Figure 3:** AIB1 regulates E-cadherin expression through E-box-dependent transcription. (A) Western blot analysis of E-cadherin and N-cadherin levels in T47D and MCF-7 cells that overexpressed AIB1 or had AIB1 knockdown. Cells were transfected with either empty vector (pcDNA) or AIB1, or with the negative control scrambled shRNA (NC) or shAIB1#1 (in the case of AIB1 knockdown). Western blot analysis was carried out using cell extract and antibody against AIB1, E-cadherin, N-cadherin or β-actin. (B) Immunofluorescence study showing the regulation of AIB1 on the expression of E-cadherin and N-cadherin. Cells overexpressed AIB1 and empty vector or AIB1 knockdown and negative control scrambled shRNA (NC) were cultured in the chamber slide and fixed, immunostained with anti-E-cadherin and anti-N-cadherin antibodies followed by the secondary antibody, Texas-red Fluor 589 anti-Rabbit. Nuclear protein was stained with DAPI. (C) Fluorescence microscopic images showing the morphology of T47D and MCF-7 cells that overexpressed AIB1 and the empty vector pEGFPC1. (D) RT-PCR analysis showing the regulation of AIB1 on the transcription of E-cadherin. The mRNA level of E-cadherin was expressed relative to GAPDH transcript level. (E) AIB1-regulated E-cadherin luciferase reporter activity. T47D cells were co-transfected with the E-cadherin-Luc reporter vector (pGL3-Ecad) and AIB1 or empty vector. Cells were harvested 48 h after transfection and subjected to luciferase activity assay. (F) Dependence of AIB1-suppressed E-cadherin transcription on E-box as shown by luciferase reporter activity. T47D cells were cotransfected with empty vector (pcDNA) or vector plus AIB1 insert (pcDNA-AIB1) together with the E-box wild-type (pGL3-Ecad) or E-box mutant (pGL3-Ecad-mut) E-cadherin-Luc reporter. Cells were harvested 48 h after transfection and subjected to luciferase activity. Relative luciferase activity was normalized to β-galactosidase activity, used as control to monitor the transfection efficiency. Each experiment was performed in triplicates and repeated at least three times. Data are the means ± SDs. Statistically significant differences (*P*<0.05) in paired Student’s t-test are marked with an asterisk.

Repression of E-cadherin transcription by AIB1 might be dependent on the presence of E-box in the promoter of E-cadherin. This was investigated by comparing the luciferase activity of T47D cells that over expressed AIB1 and E-cadherin-promoter-driven luciferase, in which the E-cadherin promoter contained wild-type E-box, and comparing it to the luciferase activity of T47D cells that overexpressed AIB1 but luciferase driven by E-cadherin promoter containing mutant box. The result showed that the level of luciferase activity obtained from wild-type E-cadherin promoter was only 25% the level obtained from the mutant E-cadherin promoter (Fig. 3F). In the case of wild-type E-cadherin promoter, overexpression of AIB1 also led to some but significant increase in luciferase activity compared to control cells (not overexpressing AIB1), whereas in the case of mutant E-cadherin promoter, no difference in luciferase activity was detected between cells that overexpressed AIB1 and control cells. Thus repression of E-cadherin expression by AIB1 required a functional E-box in the E-cadherin promoter.

### AIB1 Potentiates ERα-mediated SNAI1 Expression

EMT repressors such as SNAI1, SNAI2 and ZEB1 are implicated in E-box-dependent transcriptional repression of E-cadherin [28], and since AIB1 could repress E-cadherin expression it may achieve this through interacting with these transcription factors. Analysis of the levels of SNA1 and ZEB1 mRNAs in T47D cells that overexpressed AIB1 showed that only the level of SNAI1 mRNA was increased, reaching 2.5 fold the level of control cells, but the level of SNAI1 mRNA in AIB1-knockdown cells was reduced by 40% compared to control cells (Fig. 4A). Increases in SNAI1-promoter-driven luciferase activity in T47D cells that overexpressed AIB1 also occurred, and in a dose-dependent manner (Fig. 4B). These results indicated that AIB1 regulated SNAI1 expression at the transcriptional level.

**Figure 4:** AIB1 induces SNAI1 expression. (A) RT-PCR analysis showing the regulation of the expression of EMT-inducing transcription factor by AIB1. The mRNA levels of three EMT-inducing transcription factors, SNAI1, SNAI2 and ZEB1, in T47D cells without (pcDNA) or with AIB1 overexpression (AIB1) or without (NC) and with AIB1 knockdown (shAIB1#1) were measured by RT-PCR. The mRNA levels of SNAI1, SNAI2 and ZEB1 are expressed relative to GAPDH transcripts. (B) AIB1-regulated SNAI1 luciferase reporter activity. T47D cells were cotransfected with SNAI1-Luc and different amounts (0.1–0.5 ng) of pcDNA-AIB1 construct. Luciferase activity level in cells transfected with the empty vector pcDNA was set to 1. (C) Regulation of the activity of SNAI1 promoter by different transcription factors without and with AIB1 overexpression. T47D cells were transfected with SNAI1-Luc reporter construct and the transcription factor Sp1, ERα, E2F or Jun-D construct with or without AIB1 construct. (D) Regulation of the activity of SNAI1 promoter by nuclear receptors without and with AIB1 overexpression. T47D and HEK293T cells were transfected with SNAI1-Luc reporter vector with ERα or AR construct with and without AIB1 construct. (E) Effect of hormone and nuclear receptor inhibitor on AIB1-regulated *SNAI1* activity. T47D cells were transfected with SNAI1-Luc reporter construct with or without AIB1 knockdown, and cells were then treated with 20 nM E2 or 10 nM ICI (inhibitor of estrogen receptor) or without treatment (control) for 12 h. The levels of luciferase were normalized to β-galactosidase activity, used to evaluate transfection efficiency. Each experiment was performed in triplicates and repeated at least three times. Data are the means ± SDs. Statistically significant differences (P<0.05) in paired Student’s t-test are marked with an asterisk.

The 2-kb SNAI1 promoter region used to drive the luciferase activity (SNAI-luc construct) contains binding sites for ERα, Sp1, Jun-D, E2F as predicted by TESS: Transcription Element Search System. Some of these transcription factors have been shown to regulate SNAI1 promoter activity [7]. In order to identify which of these transcription factors might interact with AIB1, T47D cells were transfected with SNAI1-luc reporter, AIB1 and either Sp1, ERα, Jun-D or E2F. The levels of SNAI1-driven luciferase activity in cells that overexpressed Sp1, Jun-D or E2F along with AIB1 did not increase compared to cells that did not overexpress AIB1 (Fig. 4C), suggesting that AIB1 did not play a role in the regulation of SNAI1 expression by these transcription factors. In contrast, the level of luciferase activity in cells that overexpressed both ERα and AIB1 increased to more than 2-fold the level of cells that overexpressed ERα only (Fig. 4C), indicating that the combined action of ERα and AIB1 could promote the activity of SNAI1 promoter further. In addition, T47D cells that overexpressed AR (androgen receptor, which is another NR family member) together with AIB1 had higher level (40% more) of SNAI1-drive luciferase activity compared to cells that overexpressed AR only (Fig. 4D). Comparable increases in SNAI1-drivern luciferase activity were observed for HEK293T cells that overexpressed AIB1 and AR versus those that overexpressed AR only, indicating that increase in the level of SNAI1 promoter activity was not affected by the high level of endogeneous ERα as in the case of T47D cells, since HEK293T cells do not have a high level of endogenous ERα compared to T47D cells. T47D cells in which AIB1 was knocked down showed reduced SNAI1-driven luciferase activity compared to control cells (no AIB1 knockdown). However, compared to untreated cells, cells treated with E2 exhibited no change in the level of luciferase activity, but cells treated with the ERα inhibitor, ICI, exhibited almost 50% reduction in luciferase activity (Fig. 4E). This tends to suggest that ERα might regulate SNAI1 activity through coorperation with AIB1 as well as independent of AIB1. When the endogenous AIB1 of the cells was retained, treatment of the cells with E2 caused some increase in SNAI1-driven luciferase activity when the cells were treated with E2, while treatment of the cells with ICI caused some decrease in luciferase activity, but both were not significant (Fig. 4E). Thus much of the activity of SNAI1 induced by AIB1 did not appear to be contributed by the co-action of ERα, and hence E2 responsive, since the inhibition of ERα by ICI only caused slight reduction in SNAI1 activity.

### AIB1 Cooperates with ERα to Activate SNAI1 Transcription

The relevant section of the SNAI1 promoter showing the locations of ERα-binding sites and E-boxes is schematically shown in Figure 5A. To obtain further information regarding the regulation of SNAI1 promoter activity by AIB1 and ERα we used ChIP assay to analyze the region of the SNAI1 promoter that interacted with AIB1-ERα. The results revealed that AIB1 and ERα specifically associated with regions A but not with region B or C (Fig. 5B). The 2-kb SNAI1 promoter region contained multiple ERα-binding sites and E-Boxes, and three primer pairs were designed to amplify regions represented by A, B and C along the promoter as depicted in Fig. 5A. To further examine the effect that each of the regions (A–C) has on SNAI1 activity, three different truncated forms of the promoter (Fig. 5A) were constructed and each was fused to a luciferase gene to yield a reporter construct. From the ChIP assay data, it could be inferred that among the three truncated SNAI1 promoters, AIB1 specifically associated with SNAI1-a(−1061/+108), which contained regions A, B and C, and therefore all the ERα-binding sites and E-Boxes. AIB1 did not associated with SNAI1-b(−497/+108), which contained only regions B and C, or with SNAI1-c(−227/+108), which contained only region C. This suggested that AIB1 was recruited to the ERα-binding sites and E-Boxes within region A of the SNAI1 promoter (Fig. 5A), and this could be the region where ERα would actually bind to and activate SNAI1 transcription. This was subsequently confirmed by reporter gene assay, in which T47D cells transfected with the *luc* gene fused to SNAI1-a exhibited significant increase in luciferase activity when the cells over expressed either ERα, AIB1 or ERα and AIB1 compared to control cells (transfected with SNAI1-a-luc and pcDNA only) (Fig. 5C). Increases in luciferase activity over control cells were about three fold, five fold and seven folds, respectively, for cells that overexpressed ERα, AIB1, and both ERα and AIB1. No significant increase in luciferase activity was observed for cells that overexpressed AIB1 or ERα alone or together compared to control cells when the *luc* gene was fused to SNAI1-b or SNAI1-c. However, within the control cells, the level of luciferase activity was highest when the *luc* gene was fused to SNAI1-c, being almost three fold the level exhibited by SNAI1-a, and four fold the level of SNAI1-b. This suggested that SNAI1-b might contain only elements that are associated with the suppression of its activity whereas SNAI1-c probably contained no regulatory element, and the reporter activity observed was a result of unregulated threshold expression. Taken together, these results indicated that AIB1 promoted ERα-medicated SNAI1 transcription mainly via the region A of the SNAI1 promoter, which contained the first groups of ERα-binding sites.

**Figure 5:** AIB1 regulates ERα-mediated SNAI1 expression. (A) Schematic illustration of ERα-binding elements in SNAI1 promoter. Fragments A to C were chosen for PCR amplification in ChIP assays. Three truncated versions of the SNAI1 promoter were made, and the length of each is shown in the illustration. (B) ChIP assays showing AIB1- and ERα-SNAI1 promoter interaction in T47D cells. Cross-linked chromatin was extracted from T47D cells and subjected to immunoprecipitation with anti-AIB1, anti-ERα or control IgG, and the resulting precipitated DNA was used as template for PCR-ampαlification of SNAI1 promoter using specific primer covering region A, B or C of the promoter region. (C) Reporter gene assays of different truncated versions of SNAI1 promoter in the presence of AIB1 or ERαoverexpression. Each of the truncated SNAI1 promoters was fused to luciferase gene in pGL3 and the resulting construct was introduced into T47D cells along with AIB1 or ERα construct or both. The levels of luciferase activity in these cells were determined 48 h after transfection. Luciferase activity was normalized to β-galactosidase activity, used to evaluate transfection efficiency. Each experiment was performed in triplicates and repeated at least of three times. Data are the means ± SDs. Statistically significant differences (*P*<0.05) in paired Student’s t-test are marked with an asterisk.

### SNAI1 Mediates the Role of AIB1 in Promoting Breast Cancer Cell EMT

The data obtained from the preceding experiments suggested that in breast cancer cells AIB1 may suppress E-cadherin expression and promote EMT through upregulation of SNAI1. For T47D cells overexpressing AIB1, the level of SNAI1 expression was markedly reduced, at least by more than 50% (at both mRNA and protein levels) in cells with SNAI1 knockdown compared to control cells (Fig. 6A). The higher level of SNAI1 expression caused by overexpression of AIB1 was also supported by the lower SNAI1 expression in T47D cells that did not overexpress AIB1, but without SNAI1 knockdown. As for E-cadherin, the transcript and protein levels were both reduced by more than 50% in SNAI1-knocked down T47D cells that overexpressed AIB1, compared to cells that did not overexpress AIB1, with or without SNAI1 knockdown, and this reaffirmed that the difference in E-cadherin expression was caused by AIB1 (Figs. 6A&6B). These data again demonstrated that AIB1-induced EMT was dependent on SNAI1 activation, which also affected E-cadherin expression.

**Figure 6:** SNAI1 mediates the role of AIB1 in breast cancer cell EMT. (A) Western blot analysis showing the reversion of repressed E-cadherin expression in SNAI1-knockdown cells by overexpression of AIB1. T47D cells without or with SNAI1 knockdown were transfected with AIB1 and the levels of SNAI1, E-cadherin and β-actin in the cells were analyzed by western blot using the corresponding antibodies. For comparison, the levels of these proteins in T47D cells without SNAI1 knockdown and AIB1 overexpression were also analyzed. (B) RT-PCR analysis showing the level of SNAI1 or E-cadherin transcript in the different groups of cells in A. The mRNA levels of SNAI1 and E-cadherin are expressed relative to GAPDH transcripts. (C) Effect of SNAI1 knockdown on cell motility in T47D cells. The cell motility of T47D cells without or with SNAI1 knockdown that over expressed AIB1 were evaluated by scratch wound healing assay. The motility of cells without SNAI1 knockdown and AIB1 overexpression was also evaluated for comparison purpose. (D) Effect of SNAI1 knockdown on cell migration and invasion abilities of T47D cells. T47D cells without or with SNAI1 knockdown that over expressed AIB1 were subjected to transwell migration and invasion assays. Cells that migrated through the uncoated filter or invaded the Matrigel-coated filters of the chamber were detected by fluorescence imaging. The graph shows the actual number of migrated and invaded cells for each group.

In addition, scratch wound healing and transwell assays demonstrated that T47D cells with SNAI1 knockdown that overexpressed AIB1 showed reduced cell motility and invasion compared to cells without SNAI1 knockdown, but did not overexpress of AIB1 (Figs. 6C& 6D). The levels of cell motility and invasion exhibited by these cells were similar to cells without SNAI1 knockdown and AIB1 overexpression, suggesting that as in AIB1-induced EMT, which depended on SNAI1 activation, AIB1-induced cell motility and invasion also depended on SNAI1 activation.

The relevance of our findings to human breast cancer was validated by analyzing the levels of AIB1, SNAI1 and E-cadherin proteins in the invasive front of human ERα-positive breast tumor tissues. AIB1 protein level was aberrantly upregulated in invasive tumor cells, whereas SNAI1 protein level was moderately upregulated and E-cadherin protein level was downregulated in these cells (Fig. 7A). Significant correlation was observed between AIB1 and SNAI1 as well as between AIB1 and E-cadherin when the levels of these proteins in 31 ERα-positive-primary invasive breast tumor samples were compared. Although only 58% of the samples displayed high level of AIB1, 72% of these also displayed high level of SNAI1 with no detectable E-cadherin expression (Fig. 7B), which is in agreement with our speculation that AIB1 synergistically induced SNAI1 expression and E-cadherin repression, resulting in induction of EMT in the progression of breast cancer.

**Figure 7:** Correlation between AIB1/SNAI1 expressions and E-cadherin expression in human breast tissue samples. (A) Representative results of immunohistochemistry of AIB1, SNAI1 and E-cadherin in serial sections of primary tumor and invasive tumor tissues (n = 31) respectively. Each sample was incubated with antibody against ERα, AIB1, SNAI1 or E-cadherin. Positive staining and negative staining are indicated by brown and blue staining, respectively (×400 Magnification). (B) Association between AIB1/SNAI1 expressions and E-cadherin proteins in ERα+ breast cancer tissue samples. Fisher exact test, *P*<0.0001.

## Discussion

AIB1 belongs to the p160 family of transcriptional coregulators, and it interacts with nuclear receptors ERα and other specific transcription factors, forming complexes that will recruit chromatin remodeling and other transcriptional proteins to facilitate the assembly of general transcription factors, eventually leading to the transcriptional activation of many genes [15]. Moreover, high levels of AIB1 are also associated with poor prognosis in breast cancer. Although AIB1 has multiple functions, a role of AIB1 in the onset of distant metastasis is still unclear.

In this study, we found that AIB1 could control the morphological characteristics of a cell and cell-cell contact. Our results showed that knockdown of AIB1 in T47D cells increased cell-cell adhesion and induced epithelial-type morphology. Furthermore, cells treated with EGF or E2 showed a scattered distribution, and although the expression of AIB1 and ERα did not show any significant upregulation, more AIB1 existed in the form of complex with ERα (Figs. 1D&E), and AIB1 deficiency attenuated E2 signaling by reducing the ERα-activated SNAI1 promoter activity (Fig. 4E)**.** Overexpression of AIB1 in T47D cells promoted significant cell motility and invasion, but had only a slight effect on cell proliferation within 24 h (Fig. 2). Although we have shown here the importance of AIB1 overexpression and its subsequent effect on SNAI11/E-cadherin expressions, which ultimately impacted on cell motility and migration, we cannot rule out other factors that may also contribute to these two aspects and at the same time, may also be connected to AIB1 overexpression. For example, AIB1 overexpression has been shown to increase the level of IGF (insulin-like growth factor) and production of other cytokines that promote migration and metastasis [20], [29]. AIB1 amplification is known to be associated with breast tumors, especially for ERα-positive breast cancers [30], and ERα-regulated gene expression is in part dependent on the recruitment of coregulators such as AIB1 [27], [31]. Thus aberrant expression of AIB1 in a cell is likely to play a major role in controlling the morphological characteristics of the cell.

Tumor cell EMT is associated with increased cell migration, invasion, and metastasis. The well-established hallmark of EMT is the loss of E-cadherin, which disrupts the stable cell-cell adhesion between epithelial cells. Apart from E-cadherin, there is so far no other EMT inducer that has been reported. Our data showed that AIB1 expression inversely correlated with E-cadherin expression, suggesting that AIB1 may promote EMT through inhibition of E-cadherin expression, probably through interacting with the whole E-box in the proximal promoter. If transcription of E-cadherin is blocked, adhesion molecules such as N-cadherin, which has E-box in the intron, are induced during metastatic progression. In our study, the expression of N-cadherin was also increased in cells (MCF-7 and T47D) that overexpressed AIB1 (Figs. 3A&B). Expression of N-cadherin has been shown to be induced by TWIST in prostate cancer cell [32], although *TWIST* mRNA level in T47D cells was not affected by overexpression of AIB1 and ERα (data not shown). This may imply that AIB1 might regulate N-cadherin expression through other proteins or transcription factors, and this will be a subject of future investigation.

The expression of E-cadherin is subject to regulation by Snail, which functions as a transcriptional repressor, and is the most widely studied effector of EMT and E-cadherin expression. AIB1 could regulate the expression of SNAI1, but not of SNAI2 and ZEB1, probably through the ERα-binding sites located at −1061 to −790 bp of the SNAI1 promoter (Figs. 5B&C), where the ERα-AIB1 complex could bind, leading to subsequent activation of gene expression. Interestingly, the loss of these ERα-binding sites and presumably the E-box at −594 bp (SNAI1b, Fig. 5B) resulted in inhibition of SNAI1-reporter activity, whereas additional truncation that resulted in the loss of ERα-binding sites at −594 to −388 bp (SNAI1c, Fig. 5B) resulted in increased SNAI1-reporter activity. This seemed to suggest that the sequence within the −594 bp region of SNAI1 promoter may contain binding sites for repressors, and loss of this region would result in deregulation of SNAI1 expression. Conceivably, AIB1 may also enhance SNAI1 expression through other transcription factors and future investigation is required to identify these unknown transcription factors.

As for the lack of change in reporter activity observed when AIB1 was coexpressed with SNAI2-luciferase or ZEB1-luciferase in T47D cells, we could only speculate that AIB1 either did not interact with these genes in the regulation of E-cadherin expression or that additional accessory proteins or transcriptional factors are needed, which also need to be overexpressed to produce noticeable changes in the corresponding luciferase activity. Besides inhibiting the expression of E-cadherin (Figs. 6A&B), SNAI1 also been shown to inhibit the expression of epithelium-specific genes such as PTEN, Muc1, and some nuclear factor receptors [33], and in addition to its association with tumor metastasis, SNAI1 is also associated with other cancer hallmarks such as p53.

Finally, this study addressed what effect SNAI1 may have on the mammary tumor cells by acting as a target gene of AIB1. Knockdown of SNAI1 in AIB1-overexpressing T47D cells increased E-cadherin expression and decreased cell invasion capability. This appeared to suggest that upregulated SNAI1 expression was the major effect exerted by AIB1 on SNAI1 in controlling cell morphology and invasiveness. Aberrant AIB1 expression followed by SNAI1 activation and repression of E-cadherin were clearly detected at the tumor invasive front in invasive breast cancer tissue (Fig. 7A). A positive connection between AIB1 and SNAI1 expressions in breast cancer was detected since 72% of the samples with high level of AIB1 also had high level of SNAI1, although 9.6% of the samples with low AIB1 expression also had high level of SNAI1 (Fig. 7B). Furthermore, samples that showed high levels of AIB1 and SNAI1 expression also had no detectable level of E-cadherin. From a clinical perspective, since AIB1 can regulate SNAI1/E-cadherin expression, which is an important factor in tumor invasiveness, AIB1 could therefore be considered as potential marker for detecting the malignancy likelihood of breast tumor.

Short-term expression of either AIB1 or SNAI1 at moderate levels was not sufficient to induce complete EMT of human breast tumor cell line T47D cultured in vitro. This could be due to the lack of *in vivo* tumor progression environment or insufficient time for completing EMT. Furthermore, in addition to AIB1, several other coactivators have been implicated in breast cancer metastasis. For example, AIB1 can increase the function of Ets (E-twenty six) family transcription factors PEA3, AP-1 and E2F1, the activity of the IGF1 signaling pathway, epidermal growth factor (EGFR) and ERBB2, and the expression of MMPs to promote breast-tumor cell proliferation, migration, invasion and metastasis [20], [23]. Targeting AIB1 may help to reduce the extent of tumor metastasis, but since AIB1 is merely one of the genes that is associated with tumor development and progression, further study into the mechanism of AIB1-SNAI1 interaction and the identification of genes whose products are directly involved in cell motility and invasiveness will shed more light on tumor proliferation and metastasis.

## Materials and Methods

### Cell Culture and Experimental Reagents

Human breast cancer cell line ZR-75-1, MCF7 and T47D have been used in our previous study [24], [34], [35]. ZR-75-1 and MCF7 cells were cultured in Dulbecco’s modified Eagle’s medium (DMEM) containing 10% fetal bovine serum (Hyclone, Logan, UT), whereas T47D cell cells were cultured in RPMI-1640 Medium containing 0.2 Units/ml bovine insulin, 10% fetal bovine serum, 100 µg/ml penicillin and 100 µg/ml streptomycin at 37°C in the presence of 5% CO_2_. Anti-AIB1, anti-SNAI1, anti-N-cadherin, anti-β-actin and anti-ERα antibodies were obtained from Santa Cruz (Santa Cruz, CA). Anti-E-cadherin antibody was obtained from Cell Signaling (Boston, MA). EGF was obtained from Peprotech (Rehovot, Israel), and 17β-estradiol was obtained from Abcam (Cambridge, UK).

### Plasmid Construction

Human SNAI1 (Gene ID 6615) was amplified from a human cDNA library by RT-PCR and then cloned into the expression vector pEGFPC1. Human AIB1 was obtained from Dr. Anna T. Riegel (Georgetown University Medical Center, USA). The promoter regions of human SNAI1 and E-cadherin were amplified from human genomic DNA by PCR and each was separately cloned into the plasmid pGL3. Construct naming was based on the region of the promoter that was covered. Four truncated versions of SNAI1 promoter were constructed, and each was fused to a luciferase reporter gene. These were SNAI1-Luc (amplified by sense primer, 5′-GGGGTACCGGAAAGGTCTGGGATGT-3′ and antisense primer, 5′- CCGCTCGAGCCTGACGAGGAAAGAGC-3′); SNAI1-1061/+108 (amplified by sense primer, 5′-GGGGTACCTAACCAGGTCCCTCCTCA-3′, and antisense primer, 5′-CCGCTCGAGCCTGACGAGGAAAGAGC-3′); SNAI1-497/+108 (amplified by sense primer, 5′-GGGGTACCCCAGTGATGTGCGTTTC-3′, and antisense 5′-CCGCTCGAGCCTGACGAGGAAAGAGC-3′); and SNAI1-227/+108 (amplified by sense primer, 5′-GGGGGTACCGCGCTGCGCCAGCG-3′ and antisense primer, 5′-CCGCTCGAGCCTGACGAGGAAAGAGC-3′). E-cadherin-luc was amplified by sense primer, 5′-GGGGTACCCGAGGCAGAGTGCAGTGGCTC-3′, and antisense primer, 5′-CCGCTCGAGTGAAC TGACTTCCGCAAGCTC-3′.

### Luciferase Reporter Assay

Promoter activity was determined by a luciferase assay system, 24 h after transfection. For some experiments, T47D cells were transfected with SNAI1-promoter or E-cadherin promoter-luciferase construct and without or with AIB1, and luciferase activity of the cells was assayed 48 h after transfection. Luciferase activity was measured using Centro LB 960 Microplate Luminometer (BERTHOLD TECHNOLOGIES GmbH & Co KG, Germany).To evaluate the efficiency of transfectin, cells were co-transfected with the β-galactosidase plasmid followed by chemiluminescent assay [36].

### RNA Extract and RT-PCR

Total RNA was isolated from cultured cells using Trizol reagent (Invitrogen, Grand Island, NY) according to the manufacturer’s instructions [37]. RNA was quantified by optical density (A_260_) and stored at −80°C until used. One microgram of total RNA was reverse transcribed by oligo (dT) primer using Reverse Transcription System (TAKARA, Dalian, China). The single-stranded cDNA was amplified by PCR using specific primers: 5′-GGGGTACCATGCCGCGCTCTTTCCT-3′ (sense) and 5′-CGAGATCTTCAGCGGG GACATCCT-3′ (antisense) for *SNAI1*; 5′-CCCAAGCTTGCGGCCGCGATG-3′ (sense) and 5′-CTTCTAGATCACCGGTGCTTC-3′ (antisense) for *AIB1*; 5′-TCCATTTCTTGGTCTACGCC-3′(sense) and 5′-CACCTTCAGCCATCCTGTTT-3′ (antisense) for *E-cadherin*; 5′-GTTTCCCCCCACTCAACAGCG-3′ (sense) and 5′-TCCCTTGTCATTGGTACTGGC-3′ (antisense) for *ERα*; 5′-TCGTGCGTGACAT TAAGGAG-3′ (sense) and 5′-ATGCCAGGGTACATGGTGGT-3′ (antisense) *β-actin*. PCR was carried out for 30 cycles, with each cycle consisted of 94°C for 30 s, 54°C for 30 s, and 72°C for 30 s). The PCR products were analyzed by electrophoresis using a 1% agarose gel.

### Western Blot Analysis

Cells were washed three times with PBS and then lysed in HEPES containing 0.5% NP-40 and a mixture of protease inhibitors. The lysate was centrifuged to obtain the clear extract. An aliquot of the clear cell extract was used to determine the protein concentration using Bradford reagent. The cell lysates were resolved by SDS-PAGE using 10% gel. After electrophoresis, protein bands in the gel were transferred onto polyvinylidene difluoride (PVDF) membrane and were probed with the appropriate primary antibodies followed by the appropriate secondary antibodies. Positive bands of the blot were detected by ChemiLuminescence (ECL) regents (Pierce, Rockford, IL) [35].

### Immunoprecipitation

Cells were lysed in hypotonic buffer (0.5% NP-40, 20 mM HEPES (pH 7.9), 1 mM EDTA, 20 mM NaF, 1 mM dithiothreitol (DTT), 0.4 mM PMSF). After centrifugation at 13000× *g* for 2 min, the pellet (which contained the nuclear fraction) was extracted with a buffer containing 450 mM NaCl, 20% glycerol, 20 mM HEPES (pH 7.9), 1 mM EDTA, 20 mM NaF, 1 mM dithiothreitol (DTT), and 0.4 mM PMSF to yield the nuclear extract. Aliquot (500 µl) of the nuclear extract (containing 200–400 µg total protein) was incubated with specific antibody or with control IgG at 4°C for overnighte followed by addition of 25 µl of protein A and a further 2-h incubation at the same temperature (Amresco, Solon, OH) [38].

### RNA Interference

To create the AIB1 shRNA expression vector, the pRNAT-U6.1 vector (GenScript, Piscataway, NJ) was used for DNA vector-based shRNA synthesis. The sequences of AIB1 used for AIB1 knockdown study were 5′-TCCTGCAGTGTATAGTATG-3′ (shAIB1#1) [39], and 5′-GGTCTTACCTGCAGTGGTGAA-3′ (shAIB1#2) [40] and the sequence used for SNAI1 knockdown study was 5′-GGACAAAGGCTGACAGACT-3′ [41], and the sequence used for ERα knockdown experiment was 5′-CCGCTACTGTTTGCTCCTAAC-3′ [42]. The sequence of the negative control scrambled shRNA was 5′-GACGCTTACCGATTCAGAA-3′, which had no significant homology to human gene sequences [43].

### Immunofluorescence

Cells were cultured on coverslips and fixed in 4% paraformaldehyde for 15 min. After washing, the cells were permeabilized in PBS containing 0.5% Triton-X100 for 5 min. The cover slips were blocked with 0.8% BSA for 1 h and incubated with antibody against E-cadherin or N-cadherin at 4°C for overnight, followed by washing with PBS and further incubation with secondary antibody (Alexa Fluor 568) for 1 h. The cover slips were then washed with PBS and mounted on glass slides with mounting medium containing 4′,6-diamidino-2-phenylindole (DAPI), and examined and photographed using a Nikon TE2000-U microscope.

### Chromatin Immunoprecipitation Assays

Cells were crosslinked with 1% formaldehyde in PBS for 10 min at room temperature. Crude cell lysates were sonicated (typically, six 15-sec pulses followed by 45-sec rest periods at output 6.0) to generate 300 to 1500-bp DNA fragments. The sheared chromatin (25 mg) was diluted 1∶10 in dilution buffer (1% Triton X-100, 2 mM EDTA, 150 mM NaCl, 20 mM Tris-HCl pH 8.0) containing protein G and AIB1 antibody or rabbit IgG (as a negative control) and placed on a rolling shaker at 4°C for overnight. The immunoprecipitated chromatin was purified from the chromatin-antibody mixture and the chromatin immunoprecipitated DNA was eluted in elution buffer (50 mM Tris-Cl pH8, 01% SDS, and 10 mM EDTA). The purified DNA was subjected to PCR to amplify the promoter region using specific primers: 5′-TAACCAGGTCCCTCCTCA-3′ (sense) and 5′-ACGCGGCGACCGTTAAGA-3′ (antisense) for SNAII; 5′-GTGCTCTTGGCTAGATG-3′ (sense) and 5′-GACACCTGACCTTCCG-A-3′ (antisense) for; and 5′-GCACCTGCTCGGGGAGT-3′ (sense) and 5′-CCGCTCGAGCCTGACGAGGAAAGAGC-3′ (antisense) for; and 5′-CCGCTCGAGAGAGGCTGCTCCAAG-3′ (sense) and 5′-ACTCCAGGCTAGAGGGTCACC -3′ (antisense) for E-cadherin.

### Wound Healing Assay

Cells were seeded at a density of 3.0×10^5^ cells in 35-mm culture dish, and after 24 h, wounds were incised by scratching the cell monolayers with a 200-µl pipette tip. Photographs were taken under phase-contrast microscopy immediately and 24 h after incision.

### Transwell Migration and Invasion Assays

Transwell migration and invasion assay were performed in 24-well modified chambers precoated with (invasion) Matrigel (BD Transduction, Franklin Lake, NJ) or without precoating (migration). Cells in serum-free medium were transferred into the upper chamber. Following 48 h of incubation, the migrated cells in the lower chamber with 10% fetal bovine serum were counted in five random fields. Each assay was performed in triplicate.

### Immunohistochemical Assay

Sections of the tumors were first fixed in 10% buffered formalin. After fixing they were embedded in paraffin, and then deparaffinized and rehydrated using standard procedures. For antibody staining, antigen retrieval was performed in citrate buffer (pH 6.0, 30 min) and stained for the presence of ERα, AIB1, SNAI1 or E-cadherin using antibodies against these proteins. An immunohistochemistry kit (Maixin Bio, China) and DAB (diaminobenzidine) were used as chromagen for the antibody.

### Statistical Analysis

Data were analyzed by analysis of variance using the Student’s t-test. Values of p<0.05 were considered to indicate statistical significance.
